# Artificial Neural Network-Based Deep Learning Model for COVID-19 Patient Detection Using X-Ray Chest Images

**DOI:** 10.1155/2021/5513679

**Published:** 2021-06-05

**Authors:** Mohammad Shorfuzzaman, Mehedi Masud, Hesham Alhumyani, Divya Anand, Aman Singh

**Affiliations:** ^1^Department of Computer Science, College of Computers and Information Technology, Taif University, Taif 21974, Saudi Arabia; ^2^Department of Computer Engineering, College of Computers and Information Technology, Taif University, Taif 21974, Saudi Arabia; ^3^Department of Computer Science and Engineering, Lovely Professional University, Phagwara, Punjab 144411, India

## Abstract

The world is experiencing an unprecedented crisis due to the coronavirus disease (COVID-19) outbreak that has affected nearly 216 countries and territories across the globe. Since the pandemic outbreak, there is a growing interest in computational model-based diagnostic technologies to support the screening and diagnosis of COVID-19 cases using medical imaging such as chest X-ray (CXR) scans. It is discovered in initial studies that patients infected with COVID-19 show abnormalities in their CXR images that represent specific radiological patterns. Still, detection of these patterns is challenging and time-consuming even for skilled radiologists. In this study, we propose a novel convolutional neural network- (CNN-) based deep learning fusion framework using the transfer learning concept where parameters (weights) from different models are combined into a single model to extract features from images which are then fed to a custom classifier for prediction. We use gradient-weighted class activation mapping to visualize the infected areas of CXR images. Furthermore, we provide feature representation through visualization to gain a deeper understanding of the class separability of the studied models with respect to COVID-19 detection. Cross-validation studies are used to assess the performance of the proposed models using open-access datasets containing healthy and both COVID-19 and other pneumonia infected CXR images. Evaluation results show that the best performing fusion model can attain a classification accuracy of 95.49% with a high level of sensitivity and specificity.

## 1. Introduction

The novel coronavirus, also known as severe acute respiratory syndrome coronavirus 2 (SARS-CoV-2) [1], causes a respiratory illness called coronavirus disease 2019 (COVID-19). The virus was initially identified in Wuhan, China, in December 2019 and was found to cause a series of unknown pneumonia cases resulting in an ongoing pandemic [2]. The World Health Organization (WHO) declared COVID-19 a pandemic on March 11, 2020 [3]. The pandemic has caused a grievous crisis worldwide at the moment affecting 216 countries with more than 44 million cases and 1.1 million deaths around the world as per WHO statistics of November 02, 2020. Health systems are badly affected and have reached a point of failure due to inadequate facilities for intensive care units, even in the developed parts of the world.

Common symptoms attributed to COVID-19 fall in the category of fever, cold, cough, loss of taste, shortness of breath, and acute respiratory syndrome. Besides, other vital organs such as the liver and kidneys are likely to get affected by the virus, according to scientific evidence [4]. Generally, mild coronavirus cases recover within two weeks, and severe cases may take up to six weeks for complete recovery. The recovery time can sometimes be longer due to potential genetic mutations exhibited by the virus. As a whole, the ongoing pandemic poses a severe threat to our society and requires immediate action to mitigate its impact. Motivated by this, researchers are taking initiatives globally to assist health practitioners with cutting-edge technology to detect and possibly prevent the further spread of the virus.

Early detection of coronavirus cases is vital so that patients with the disease can be quarantined to reduce transmission. Currently, the gold standard for diagnosing COVID-19 is real-time reverse transcription polymerase chain reaction (RT-PCR), which is a laboratory-based procedure to test for the presence of SARS-CoV-2 RNA (ribonucleic acid) in a sample (more recently saliva sample) taken from the patient. Typically, a real-time RT-PCR process takes approximately 4–6 hours to obtain the test results. Furthermore, RT-PCR test kits are short in supply. Consequently, many COVID-19 patients cannot be identified at early stages and are likely to infect other people inadvertently.

To overcome the shortage of testing kits, various efforts have been undertaken to discover alternative testing methods. Generally, different radiology images such as chest X-ray (CXR) and CT (computed tomography) scans are easily accessible to health practitioners in clinical procedures. These medical imagery modalities can play a vital role in confirming the diagnosis of COVID-19 contraction and monitoring disease progression over time. Ground-glass opacities (GGOs) are abnormal patterns observed in CXR and chest CT images when the lungs are sick. According to a study [5], GGOs are commonly seen findings in patients with COVID-19 related pneumonia.

Computational models in the area of AI and deep learning have been significantly used in solving problems related to medical imaging [6, 7] and general disease identification systems [8–10]. Since the onset of the pandemic, many researchers have shown the effectiveness of using radiology images in identifying COVID-19 infection with various deep learning techniques. Owing to the shortage of publicly available big COVID-19 related image datasets, most of the existing works used limited-size training samples and are likely to face the generalizability problem to unseen data.

Lately, there has been a growing interest in developing fusion models from heterogenous technologies and explicitly training fusion networks. Multiple deep learning models (wide and deep) are combined to make superior predictions. Thus, the fusion representation of deep learning models allows us to assimilate various individual networks' strengths to achieve promising performance. To this end, we have proposed a deep learning-based end-to-end fusion model that exploits the benefit of a combination of parameters (weights) from multiple deep CNN models to expedite the testing of CXR images in the automated detection of positive COVID-19 encounters. Specifically, our approach uses the Polyak and Juditsky technique [11] to obtain an average of parameters (weights) from different models seen towards the end of the training process. These average model weights are fit into a single clone model to extract features from images, which are then fed to a custom classifier for the final classification of CXR images.

We have experimented with three different fine-tuned CNN models called ResNet50V2 [12], VGG-16 [13], and InceptionV3 [14] to observe the benefit of parameter fusion in extracting salient features from the input CXR images. Furthermore, we utilize an explain-ability method to investigate how our models make predictions to facilitate clinicians' improved diagnosis. To evaluate our proposed models, we have used a curated dataset of CXR images that are collected from two publicly available data repositories containing images from normal, COVID-19, and other non-COVID-19 pneumonia categories.

In summary, we have made the following key contributions to this paper:

- A deep learning-based CNN fusion framework is introduced for the automatic screening of COVID-19 patients using CXR images.
- Parameters (weights) from different fine-tuned CNN models are combined into a single model to extract features from images to enhance diagnosis performance.
- An explain-ability method is developed using gradient-weighted class activation mapping to visualize the infected areas of CXR images.
- A comparative study is presented to investigate the effectiveness of the proposed weight fusion model and individual base CNN models.
- We present extensive experimental analysis to demonstrate the performance of the studied models. The proposed best performing fusion model achieves an accuracy of 95.49% in classifying COVID-19 images with a high degree of precision (96.19%), sensitivity (99.19%), and AUC score (95.94%).

The remainder of the paper is structured as follows. Related studies are presented in Section 2. The proposed methodology, including the collection and preparation of the dataset, is described in Section 3. Performance results, analysis, and discussion are presented in Section 4. Finally, conclusions are presented in Section 5 with some potential future work.

## 2. Related Literature

Since the onset of the COVID-19 pandemic, researchers have proposed deep learning-based methods for automatic screening of positive COVID-19 cases using different radiology images such as CXR and CT scans. This section contains the studies related to COVID-19 diagnosis and has primarily employed various AI-based techniques, especially machine learning and deep learning.

Zhang [15] proposed a CNN-based approach to address the problem of extracting relevant and important features from limited training data. Specifically, they developed a triple-view CNN architecture for the automatic diagnosis of COVID-19 patients. They utilized three different views (left lung, right lung, and overall view) of a CXR image to extract individual features and integrate them for joint prediction. They have employed six different fusion methods based on various feature pooling and concatenation mechanisms. The performance results showed the effectiveness of their proposed model for binary classification of healthy and COVID-19 cases and three-class classification with healthy, COVID-19, and other non-COVID-19 pneumonia cases.

Ghoshal and Tucker [16] introduced a deep learning-based technique to estimate the uncertainty and interpretability in detecting coronavirus. The authors have used a Bayesian convolutional neural network (BCNN) and publicly available COVID-19 CXR images and found that the prediction uncertainty is extremely correlated with prediction accuracy. The performance results demonstrate an improvement in detection accuracy from 85.2% to 92.9% using the pretrained VGG-16 model. They have also illustrated model interpretability by generating saliency maps to better understand the results obtained by the proposed model.

Narin et al. [17] presented a transfer learning-based approach to categorizing CXR images into COVID-19 and normal categories. They have used three pretrained models, namely, InceptionV3, ResNet50, and InceptionResNetV2, in their system and achieved the highest (98%) accuracy with ResNet50 for binary classification. However, the number of COVID-19 images in the curated dataset is only 50.

In another effort, Oh et al. [18] have introduced a patch-based technique to train and fine-tune the ResNet18 CNN model. They have used patches extracted from input CXR images to train the model. A majority voting strategy was used to obtain the final classification decision, and the model attained a moderate accuracy of 88.9% in a multilabel classification scenario. Ozturk et al. [19] took an approach different from the majority of the AI-based detection models for COVID-19, where they proposed an objected detection-based technique. They have trained a DarkNet model for the classification of CXR images for COVID-19 detection. The experimental results showed a high level of accuracy (98.08%) for binary classification. However, the model exhibited relatively low performance for multiclass classification and attained an accuracy of 87.02% only.

Jain et al. [20] have used transfer learning-based techniques to detect and analyze COVID-19 cases using X-ray images. The authors compared the performance results of three pretrained CNN models, namely, InceptionV3, Xception, and ResNeXt, using X-ray images from an open-source data repository and found that the Xception model produces the highest (97.97%) accuracy. In another study, Hoon et al. [21] proposed a deep learning-based decision tree classifier for COVID-19 screening using CXR images. More specifically, they built three binary decision trees, as part of the classifier, which were trained using a convolutional neural network. The first tree classifies normal or abnormal images, while the second tree determines if the abnormal images are from the *tuberculosis* category. Finally, the third decision tree identifies COVID-19 encounters. The experimental results showed that the final decision tree could classify coronavirus cases with an accuracy of 95%.

Sharma et al. [22] used extensive image preprocessing and augmentation to increase the dataset's size and leveraged the transfer learning method for training and validating classification models. They have combined the two best performing models. Each model was trained using CXR images with a certain degree of rotation and obtained state-of-the-art detection accuracy in identifying COVID-19 cases. In a successive effort, Sakib et al. [23] suggested a deep learning-based framework that leveraged a data augmentation algorithm for radiography images. The framework adaptively used generative adversarial network (GAN) and generic augmentation techniques to produce synthetic COVID-19 images. A custom convolutional neural network model was trained with the augmented images, and an accuracy of 93.94% was obtained on the test data.

Haque and Abdelgawad [24] have proposed a custom convolutional neural network model to detect COVID-19 patients using two different datasets containing normal and COVID-19 positive images. The proposed model achieved an accuracy of 98.3% using a second dataset. However, the model has only considered binary classification, and hence it cannot differentiate between COVID-19 and other non-COVID-19 cases of pneumonia.

Waheed et al. [25] applied data augmentation based on auxiliary classifier generative adversarial network (ACGAN) to improve detection accuracy. The authors were able to increase the accuracy to 95% by using the synthetic images generated from the proposed GAN-based architecture. In another effort, Periera et al. [26] performed COVID-19 identification based on multiclass and hierarchical classification scenarios. They have applied both early and late fusion techniques in the classification schema to use hand-crafted texture features and features extracted from a pretrained CNN model. The evaluation results demonstrated the effectiveness of the proposed approach with an F1-score of 0.89 for COVID-19 identification.

Islam et al. [27] proposed a deep learning technique combining convolutional neural network (CNN) and long short-term memory (LSTM) to automatically detect coronavirus infection from CXR images. They have used the CNN model to extract salient features which are then fed into the LSTM network for COVID-19 classification. The experimental results were obtained using a dataset containing 4575 CXR images, out of which 1525 images were from the COVID-19 category. The proposed model achieves an accuracy of 99.4% with a high degree of sensitivity and specificity.

Gianchandani et al. [28] presented an ensemble of deep transfer learning models from CXR images to differentiate COVID-19, viral pneumonia, and bacterial pneumonia. They leveraged four modified transfer learning models, namely, VGG16, ResNet152V2, Inception ResNetV2, and DenseNet201, and selected the two best performing models to create the ensemble network, which was followed by two dense layers for final classification. They evaluated their model using two well-known datasets and achieved an accuracy of 99.21% for multilabel classification. In a similar effort, Singh et al. [29] employed a similar ensemble model consisting of densely connected convolutional networks (DCCNs), VGG16, and ResNet152V2 to detect COVID-19 from chest CT scans. The experimental results demonstrated the effectiveness of the proposed ensemble model in terms of all the common performance metrics, including accuracy, sensitivity, and specificity. Das et al. [30] presented a truncated Inception Net for detecting COVID-19 from CXR images. The authors employed six different types of datasets containing COVID-19, pneumonia, tuberculosis, and healthy cases for model training and testing.

Wang et al. [31] proposed a deep learning model for detecting COVID-19 patients from CXR images and achieved an accuracy of 93.3% in classifying COVID-19, pneumonia, and normal cases. Towards the beginning of the pandemic, we have proposed a deep learning model based on fine-tuned CNNs and obtained a performance accuracy of 98.15% with a small dataset [32]. However, we noticed that the model seemed to suffer from an overfitting problem with the relatively larger dataset, and the performance was somewhat degraded. To overcome this problem, we employed the parameter (weight) fusion model concept in this study. Besides, some other works focused on explainable AI [33–35], metalearning [36], and segmentation [37] based frameworks for COVID-19 and pneumonia-related healthcare systems.

Generally, deep transfer learning models used in the literature for COVID-19 detection face difficulty in converging due to their challenging training process. Hence, the final model may not be stable or may not have the best set of parameters (weights). Consequently, training and validation loss will show higher than anticipated variance and bounce up and down during the training process. To overcome this problem, we introduce a weighted fusion of parameters in our system. We take the average of the weights from multiple models of the backbone network observed near the end of the training process.

Moreover, while current deep learning approaches have shown their advantage over other techniques in COVID-19 detection, most of these approaches do not support their findings with sufficient interpretability of models related to pertinent features of pathological signs in the CXR images. Thus, the clinical efficacy of these techniques is uncertain until further studies are undertaken to interpret the high-level features extracted from these models. It is highly improbable that clinicians in real life are going to accept a black-box classification model even with highly accurate experimental results. Our proposed system provides an explain-ability method to produce heatmaps that visualize the areas of CXR images that are most indicative of the disease. This provides interpretability of our model's decision in a manner understandable to the clinicians.

## 3. Materials and Methods

We have proposed a deep learning-based fusion model that exploits the benefit of a weighted average of the model weights from backbone CNN models in extracting salient features from the input CXR images that are used to obtain a robust classification of these images into COVID-19, normal, and pneumonia categories. This section starts by describing the various components of our proposed system and the underlying technology to realize COVID-19 screening from the supplied CXR data.

Figure 1 shows the overall architecture of our proposed COVID-19 detection system, which consists of several steps. First, we create a curated dataset containing COVID-19, normal, and other pneumonia CXR images from two publicly available data sources. Original CXR images are then passed through a data preprocessing pipeline to perform various tasks such as normalization, resizing of the image, and shuffling. Different image augmentation techniques are used for model training and validation to overcome the problem of limited training data and increase model generalizability. The preprocessed image data is then split into training, validation, and test sets, from which we have used the training and validation data to train and validate our models through 5-fold cross-validation. We have performed a weighted fusion of parameters (weights) from multiple instances of backbone CNN models along the way. We have considered three widely used deep CNN models, namely, VGG-16 [13], InceptionV3 [14], and ResNet50V2 [12], as our backbone models. The performances of the proposed models are then measured with the test dataset using standard metrics.

### 3.1. Proposed System

We present a schematic diagram of our proposed system (as shown in Figure 2) to automatically detect COVID-19 cases using a weighted fusion of parameters from deep CNN models. First, we perform parameter (weight) fusion from the weighted combination of the parameters extracted from multiple backbone CNNs. The architecture of each backbone network can be either custom-designed or off-the-shelf pretrained network architecture. However, to facilitate the weight fusion mechanism, these network architectures need to be identical. A clone of the backbone architecture conducts multilabel classification on the fused parameters to realize coronavirus infected cases.

Finally, model interpretation through feature representation is demonstrated using the t-SNE visualization technique to investigate how good the feature representations obtained from the clone network. A detailed description of the system is given in the following subsections.

#### 3.1.1. Backbone Network Architecture

Our system has used the above-mentioned three pretrained (on ImageNet dataset [38]) CNN models along with their weights from convolutional layers for feature extraction from input CXR images. The VGG-16 network architecture [13] represents a simple network with only 3 × 3 convolutional layers stacked together in increasing depth. Besides, the volume size is reduced using max-pooling layers. As the name suggests, it has 16 weight layers with the last two fully connected layers, each with 4,096 nodes followed by a softmax classifier layer. Traditional sequential deeper networks such as VGG-16 suffer from the vanishing gradient problem where the accuracy becomes saturated and drops abruptly with increasing depth. ResNet architecture [12] addresses this problem by skipping through less important layers with residual modules while training the network with a standard SGD optimizer. The ResNet (ResNet50V2) version used in this study contains 50 weight layers demonstrating a significant decrease in the model's size and the number of FLOPs. The third CNN model used in our fusion network is Inception, introduced by Szegedy et al. [14]. It appears as a microarchitecture to use a multilevel feature extractor by computing convolutions of different sizes (1 × 1, 3 × 3, and 5 × 5) within the same network module. Outputs from these filters are stacked on top of each other along the channel dimension and then fed into the next layer. The original manifestation of this network was called GoogLeNet, but the subsequent incarnations are simply named as Inception with appropriate versions. In this study, we have used InceptionV3 [39], an updated version of the Inception module that achieves further improvement in ImageNet classification accuracy. InceptionV3 is characterized by its weights, which are less than those of both ResNet and VGG.

As part of fine-tuning, we delete the classifier part of the backbone CNNs. We include our custom prediction layer consisting of a GAP (global average pooling) layer followed by double dense layers consisting of 256 neurons and three neurons. As opposed to the flattening layer, a GAP layer can better address the overfitting problem by reducing the number of model parameters. In the GAP layer, an *h* × *w* feature map is converted to a single value by computing the average of all pixel values in the feature map and thus obtains 1 × 1 × *d* tensor from a 3D tensor of dimension *h* × *w* × *d*.

#### 3.1.2. Weighted Parameter Fusion

As shown in Figure 3, we carry out the fusion of parameters (weights) extracted from the backbone CNN models. This process is also known as “early fusion.” The resulting fused parameters are then fit into a clone architecture of the backbone network, which extracts features for final prediction. Thus, our fusion architecture can be treated as end-to-end, trainable, and capable of learning rich feature representations and performing multilabel classification through prediction. We introduce a weighted fusion of parameters in our system primarily motivated by the fact that deep learning models often fail to converge due to their challenging training process. This implies that the model obtained at the end of the training phase may not be stable, or the final model may not have the best set of parameters (weights). In other words, if the model faces difficulty in converging, training and validation loss will show higher than anticipated variance and bounce up and down during the training process.

To address this issue, we take the average of the weights from multiple models of the backbone network observed near the end of the training process. This is known as the Polyak averaging or Polyak–Ruppert averaging technique [11], widely used in stochastic gradient methods. It is achieved by averaging multiple points in a parameter space traversed by an optimization algorithm. If we consider that *n* iterations of a gradient descent algorithm traverse *n* points (*θ* (1), *θ* (2),…, *θ* (*n*)) in the parameter space, then we obtain the output $\left({\hat{\theta }}^{\left(n\right)}\right)$ from the Polyak averaging algorithm [11] as follows:

(1) $$\begin{array}{c} {\hat{\theta }}^{\left(n\right)}=\frac{1}{n}\underset{i}{\sum \theta^{\left(i\right)}}. \end{array}$$

For some specific problem classes, such as gradient descent applied to a convex problem, this technique shows a more robust assurance of convergence. More specifically, the optimization algorithm may switch back and forth in the valley without touching a point near the bottom of the valley. Polyak average of the visited points on either side of the valley would produce the desired result by settling a point closer to the bottom of the valley. As for the nonconvex problems, the optimization paths can be more complex and include many distinct regions. In such cases, it is beneficial to use an exponentially decaying average when applying the Polyak technique [11] to nonconvex problems as follows:

(2) $$\begin{array}{c} {\hat{\theta }}^{\left(n\right)}=\alpha {\hat{\theta }}^{\left(n-1\right)}+\left(1-\alpha \right)\theta^{\left(n\right)}. \end{array}$$

In this study, we consider equally, linearly decreasing, and exponentially decreasing weighted average of model parameters from multiple models to develop the final fusion CNN models. The detailed technique for the calculation of average model weights is described below.

Our goal is to build a new weight fusion model from multiple existing models with varying weights (parameters) with the same architecture. We can build the new model by taking the weighted average of the model weights. Convolutional layers are the primary building blocks of the CNN models. Each convolutional layer of a model contains two sets of weights: a block of filters and a block of biases. We retrieve these weights from the same layer of each model and compute the weighted average, which provides us with a new set of weights. Then, we build a clone of the base architecture and fit these calculated weights to obtain the new fusion model. Based on the three averaging techniques mentioned above, we calculate the new set of weights as follows:

For equally weighted average,

(3) $$\begin{array}{c} W_{i}=\frac{1}{n},\;1\leq i\leq n. \end{array}$$

For weighted average with linear decay,

(4) $$\begin{array}{c} W_{i}=\frac{i}{n},\;n\geq i\geq 1. \end{array}$$

For weighted average with exponential decay,

(5) $$\begin{array}{c} W_{i}=e^{-\left(i/\alpha \right)},1\leq i\leq n, \end{array}$$

where *W*_*i*_ represents the weighting factor for each of the *n* models and *α* denotes decay rate. Finally, we obtain the filter weights, *w*_*f*_, and bias values, *b*_*f*_, of the fusion model by applying *W*_*i*_ in each model's weights:

(6) $$\begin{array}{c} w_{f}=\sum_{i=1}^{n}w_{i}*W_{i},\\ b_{f}=\sum_{i=1}^{n}b_{i}*W_{i}. \end{array}$$

#### 3.1.3. Feature Representation

To support the qualitative analysis, we investigate how well the features are distributed in the feature space to understand the class separability. Since convolutional layers produce high-dimensional outputs, we need to adopt a dimensionality reduction technique to visualize them in 2D space. To achieve this, we use t-SNE (t-Distributed Stochastic Neighbor Embedding) [40], which is a popular technique for exploring and reducing high-dimensional data. t-SNE does this by calculating the affinities between data points and preserving these affinities in the reduced low-dimensional space.

Let *X* be a matrix consisting of all samples in the dataset and *Y* be a target matrix containing the low-dimensional representation. The similarity between two data points in the original high-dimensional space can be expressed as a conditional probability [40]:

(7) $$\begin{array}{c} P_{j|i}=\exp\left(\frac{-{\left\|x_{i}-x_{j}\right\|}^{2}}{2\sigma^{2}}\;\right),\;\text{normalized s}\mathrm{.t}\text{. }\forall i\sum_{k}p_{k|i}\;. \end{array}$$

The affinity metric can be obtained by using a symmetric variant of equation (1) where the affinities of U to V and V to U are the same [40]:

(8) $$\begin{array}{c} P_{ij}=P_{i|j}+P_{j|i}\text{,}\;\text{normalized s}\mathrm{.t}\text{.}\sum_{i}\sum_{j}P_{ij}=1. \end{array}$$

Similarly, the affinities in low-dimensional space are calculated considering a Student *t*-distribution for *d* dimensions as follows [40]:

(9) $$\begin{array}{c} Q_{ij}={\left(1+\;\frac{{\left\|y_{i}-y_{j}\right\|}^{2}}{d-1}\right)}^{-\left(d/2\right)},\;\text{normalized s}\mathrm{.t}\text{.}\sum_{\text{i}}\sum_{\text{j}}Q_{ij}. \end{array}$$

Given the affinities for every pair of data points in both high- and low-dimensional spaces, the goal is to keep them closer as much as possible. A loss function is used to estimate the distances between the similarities. t-SNE uses Kullback–Leibler divergence as a loss function since the similarities are defined using probabilities [40]:

(10) $$\begin{array}{c} \text{KL}\left(P\left\|\right)Q\right)=\sum_{i}\sum_{j}P_{ij}\log\frac{P_{ij}}{Q_{ij}}. \end{array}$$

## 4. Results and Discussion

To demonstrate the efficacy of our proposed system in screening COVID-19 encounters, we extensively evaluate and compare the performance results of the model with fine-tuned transfer learning models, namely, ResNet50V2, VGG-16, and InceptionV3, using two publicly available CXR datasets.

### 4.1. Dataset Preparation

We have collected CXR images from two open-source repositories. First, a total of 616 COVID-19 positive images are gathered from the GitHub repository managed by Cohen et al. [41]. Second, we collected the same number of normal and other non-COVID-19 pneumonia images from the Kaggle repository [42] to avoid class imbalance in the curated dataset. Thus, the final dataset contains a total of 1848 X-ray images comprising all three classes: healthy, COVID-19, and other non-COVID-19 pneumonia. To assess the used models' performance, we have used a 5-fold cross-validation technique where the entire dataset is divided into five equal parts at the patient level.  Table 1 shows the distribution of images at a ratio of 60 : 20 : 20 in each fold for training, validation, and test datasets. We use the training and validation sets during training, while the holdout test set is used to evaluate the models.

The CXR images in the curated dataset come in varying sizes due to different clinical settings. We have performed several fundamental preprocessing tasks to prepare the input images suitable for model training and validation. All images are resized to 224 × 224 pixels, and all pixel values are rescaled to [0, 1] through the min-max normalization technique. Some CXR image samples from different categories are shown in Figure 4. A healthy CXR image exhibits clear lungs and does not contain any irregular “opacification” area. Bacterial pneumonia typically displays a focal nonsegmental pattern shown with white arrows in the upper right lobe in the image. On the contrary, viral pneumonia tends to show a narrow “interstitial” pattern in both lungs. Finally, patients with COVID-19 infection mostly show multifocal and bilateral ground-glass opacities in the CXR images [43]. Besides, we use image augmentation to tackle the problem of a small dataset and increase training efficiency while preventing the models from overfitting. A summary of the augmentation features used for preparing the training dataset is given in Table 2.

### 4.2. Experimental Settings

The fine-tuned CNN backbone models and the proposed parameter fusion model are implemented using TensorFlow. More specifically, we have used Keras functional API to build the fusion model, which can handle models with shared layers, nonlinear topology, and multiple inputs or outputs. We also use a special form of model cloning from Keras to implement the fusion model with updated average parameters (weights), which has the same architecture as the backbone network. We use the Google Colab environment for the implementation of all our models. Colab offers free GPU access, which is crucial for training deep learning-based computer vision models. It comes with all necessary Python 3.x packages preinstalled with Keras API and TensorFlow backend. Towards the end of the parameter fusion architecture, we add a dense layer with 256 neurons with the ReLU activation function. Lastly, a fully connected layer with a softmax activation function is added to produce the classification scores.

We start model training with an initial learning rate of 0.001. Then, the learning rate is adjusted with decay computed from the ratio of the initial learning rate to the number of training epochs. Moreover, Keras callback called ModelCheckpoint is used to monitor the performance metrics and periodically save the model based on some monitoring criteria such as validation loss or accuracy. We have used accuracy, precision, sensitivity, specificity, F1-score, and AUC (area under curve) as our performance metrics.

### 4.3. Result Analysis

We start by investing the learning curves obtained by all backbone models without any parameter (weight) fusion during training and validation. All the models show a modest learning progression (as shown in Figure 5) during the training period by incurring a relatively unstable decline in both types of losses. This implies that the model obtained at the end of the training phase may not be stable, or the final model may not have the best parameters (weights). In other words, the tested models show higher than anticipated variance, and training and validation losses bounce up and down during the training process. We take the weights from multiple models of these backbone networks observed near the end of the training process (approximately the last 10 epochs) to address this issue. The updated weight is then fit to a clone model obtained from each of them.

As stated earlier, we have considered three variants of average weight calculation, such as a simple average of weights and linearly and exponentially decreasing weighted average.  Figure 6 reports validation accuracy curves of the ResNet50V2 model observed for the last eleven epochs with all three average weight types. It is evident from the performance curves that the validation accuracy scores show a more substantial stabilizing effect of employing exponential decay instead of a linear or equal weighting of models. Thus, the use of the exponential decay of model weights would be preferred over other averaging methods for the overall performance evaluation of the models.

We compare the performance results of various fusion CNN models using the holdout test dataset. In addition to the overall performance (as shown in Table 3), class-wise performance is also evaluated using the same metrics (shown in Table 4). It is noticed that the ResNet50V2 model shows consistently better results than other models in performance metrics, including accuracy (95.49%), sensitivity (99.19%), and area under the curve (AUC), which are deemed to be very critical performance estimates for applications in medical settings. The sensitivity result indicates that ResNet50V2 can accurately identify positive COVID-19 cases with an accuracy of 99.19% from all positive cases. Surprisingly, VGG-16 and InceptionV3 show values of precision and specificity superior to those of ResNet50V2.

We also present class-specific results for various models in Table 4. All the models tend to show relatively low performance in classifying pneumonia images while delivering moderate performance in identifying healthy cases. As per classifying the COVID-19 positive subjects, ResNet50V2 offers superior performance in terms of accuracy and sensitivity. This result is hypothetically meaningful since accurately classifying CXR images for all three subject groups (COVID-19, normal, and pneumonia) is essential for a useful diagnostic tool.

For a deeper understanding of the performance of the evaluated models, the receiver operating characteristic (ROC) curve and confusion matrix for each model are shown in Figure 7 and Table 5, respectively. A ROC curve plots the true positive rate (TPR) against the false positive rate (FPR). All the tested CNN models show superior discrimination abilities for COVID-19 classes but exhibit poor classification performance for non-COVID-19 types. This is substantiated by the fact that the curve for COVID-19 is slightly higher than the other classes. We observe from the confusion matrix (in Table 5) a reduced count of FN cases for ResNet50V2, which implies that the number of COVID-19 cases that are missed is less, and it contributes to an increased value of sensitivity. In reality, it is vital to keep the count of FN cases low and ensure that the model does not identify somebody contracted with the virus as healthy, thus hampering the patient's line of treatment. However, we observe that both VGG-16 and InceptionV3 models generate fewer false positive (FP) cases for COVID-19 classes than ResNet50V2.

FP's low value indicates that the number of cases that are misidentified as COVID-19 positive is less and positively contributes to increased values of precision and specificity. To limit the count of FP cases is very important to reduce unwanted financial liabilities on health providers.

### 4.4. Visualization

Figure 8 shows the visualization of features extracted from various CNN models using CXR images from the holdout test dataset. It is observed that the ResNet50V2 model exhibits better feature representation compared to other models. The t-SNE of all the fusion models seems to be well-plotted in a relatively compact space and shows a clear separation of COVID-19 classes compared to normal and pneumonia classes. However, all the models show an area of overlap between normal and pneumonia classes.

We also investigate how the models are making decisions regarding COVID-19 prediction. It is crucial to comprehend what the models are learning from the input images during training and validation [44, 45]. We use Grad-CAM [44], which works based on the gradients with respect to the target class flowing into the last convolutional layer to generate a localization map pinpointing the crucial regions in the image for correct prediction.

Figure 9 shows the heatmap visualization of two CXR images of both COVID-19 and other pneumonia patients with Grad-CAM. The illustration includes the original image (focus areas marked with red arrows in the second image) followed by a heatmap highlighting the critical regions within the lungs and an overlay of heatmap onto the original image using ResNet50V2 and InceptionV3. ResNet50V2 seems to focus on both sides of the respiratory tract to classify this particular case. However, InceptionV3 seems to focus on relatively larger areas, including the lower respiratory tract, even though both the models have produced correct predictions for the image. This needs to be verified clinically with an experienced radiologist through careful testing. The bottom line is to make sure that our model depends on proper knowledge from the images to make the classification decisions.

### 4.5. Discussion

To summarize, we have presented the performance comparison between the proposed fusion models in this study to detect COVID-19 cases automatically. Based on the presented results, we conclude that our fine-tuned weight fusion model using ResNet50V2 appears to be the best performing model. It is worthwhile to mention that the size of the dataset used in this study containing COVID-19 CXR images is still limited and merely adequate to train our proposed fusion models to obtain stable classification performance. Hence, one of our future goals is to collect more COVID-19 images as they become available to ensure that the curated dataset contains sufficient training and validation data and thus overcome the data scarcity problem. With more data, we expect that our model will achieve further improvement in prediction results.

We also compare our proposed fusion model with a representative set of existing studies from the literature. As such, the comparison results are presented in Table 6. It is worth noting that the size of the CXR dataset used in some of these studies with COVID-19 positive cases is very small. For model training, some of the earlier studies (e.g., [17, 31]) used even less than 100 COVID-19 images. Wang et al. [31] proposed COVID-Net as one of the first attempts to detect COVID-19 from CXR images. For the prediction of COVID-19 events, they proposed a custom deep learning model. However, the model training dataset includes less than 100 COVID-19 samples and a significant number of samples from the healthy and non-COVID-19 groups. As a result, their dataset is a bit unbalanced, which could affect the model's performance. Narin et al. [17] used several pretrained transfer learning models and achieved the highest accuracy of 98% with ResNet50 for binary classification. However, there are only 50 COVID-19 images in the curated dataset that they used. Waheed et al. [25] addressed the issue of limited training data by generating synthetic images using generative models and achieved an accuracy of 95%. However, their approach suffers from a high false negative rate. Although the false predictions in ResNet18 [18] and Dark COVID-Net [19] are relatively less, the model accuracy is only 88.9% and 87%, respectively, for the multiclass classification problem. The triple-view CNN architecture proposed by Zhang [15] achieved high accuracy (99.8%) for binary classification of healthy and COVID-19 cases but showed comparatively lower performance in terms of accuracy (84.4%) for three-class classification with healthy, COVID-19, and other non-COVID-19 pneumonia cases. The deep learning-based decision tree classifier proposed by Hoon et al. [21] showed a similar performance to our proposed fusion model, where the final decision tree could classify coronavirus cases with an accuracy of 95%.

Based on the above discussion, we observe that the proposed fusion model shows performance similar to or better than many other existing studies in terms of accuracy, sensitivity, specificity, and AUC in detecting COVID-19 cases considering a 3-class classification problem. Given the amount of work done so far for the automatic diagnosis of COVID-19 patients using deep learning models, we can realize AI's role in assisting health practitioners for proper and faster diagnosis of this deadly virus during the ongoing pandemic. This research is one step near a more transparent comprehension of the infections caused by this novel coronavirus. It proposes an improved deep learning-based solution for automatic and fast detection of potential COVID-19 encounters.

It is imperative to state some of the limitations of our current work. Research findings from some recent studies suggest three distinct stages of COVID-19 disease progression: early infection, pulmonary phase, and hyperinflammation phase [46]. Each of these stages shows variable degrees of symptoms. The early infection phase is characterized by mild symptoms such as common cold or flu. In the pulmonary phase, the infection strongly affects the patient's immune system with primary respiratory symptoms, including frequent cough, shortness of breath, and reduced oxygen levels. In the third stage, patients develop acute respiratory distress syndrome (ARDS) and may experience injury to kidneys and other organs. Our proposed model cannot identify the stage at which the disease is detected from the CXR images. Further study is required with appropriate metadata along with the CXR images to report the exact stage of disease in addition to mere diagnosis. In addition, our work is limited by the fact that the curated dataset is composed of CXR images (COVID-19, normal, and other non-COVID-19 pneumonia) from two different sources. A critical study by Maguolo and Nanni [47] reveals that this heterogeneity of data sources might add a bias to the prediction. Hence, the learning patterns of the model might not entirely be correlated to the existence of COVID-19.

Although recent findings suggest that CXR images may not be the best modality for early detection of COVID-19, other research findings (reported in the literature studies) confirm that radiology images show salient information about COVID-19 infection during disease progression. Thus, we would safely argue that our proposed fusion model is by no means a replacement for a human radiologist. Instead, we expect our current findings to offer a valuable contribution to the growing recognition and adoption of AI-aided applications in clinical settings. Even if it is not sufficient to solely rely on the results obtained from CXR images to prescribe the line of treatment for a patient, an automated early screening can greatly help health professionals identify and quarantine positive encounters until a comprehensive test is conducted.

## 5. Conclusions and Future Work

In this paper, we introduce a novel CNN-based deep learning fusion framework using the transfer learning concept to detect COVID-19 from CXR images automatically. The fusion architecture takes the average of the weights from multiple models of the backbone network observed near the end of the training process and fits them to a single model to extract features from images, which are then fed to a custom classifier for prediction. Specifically, we use ResNet50V3, VGG-16, and InceptionV3 models and leverage the models' weighted contribution with exponential decay to improve the performance. The best performing model (ResNet50V2) obtains an accuracy of 95.49%, sensitivity of 99.19%, F1-score of 98.0%, and AUC of 95.49%. Our model also shows desirable explain-ability properties by efficiently identifying various areas in CXR images related to COVID-19 infection. We anticipate that the results achieved from our proposed fusion model will assist clinicians in the automatic detection of COVID-19 patients and reduce their workload. Simultaneously, it is important to identify some of the limitations of our work, which could be addressed in future studies. The major drawback is that the dataset used in this analysis, which contains COVID-19 CXR images, is still limited. As an immediate future work, we plan to extend our work by collecting more COVID-19 images as they become available to achieve further improvement in prediction results. In the future, we also plan to adopt an improved fusion model based on feature concatenation extracted from CXR images and multimodal COVID-19 data for enhanced prediction results.

## Figures and Tables

**Figure 1:** Process diagram showing the development flow of our proposed system.

**Figure 2:** Schematic diagram of our proposed COVID-19 detection system with parameter fusion.

**Figure 3:** Illustration of various parameter fusion techniques in the proposed system: (a) weights from CNN models; (b) average; (c) linearly decreasing weighted average; (d) exponentially decreasing average.

**Figure 4:** Samples of CXR images from the curated dataset: (a) healthy; (b) bacterial pneumonia; (c) viral pneumonia; (d) COVID-19.

**Figure 5:** Training and validation curves for (a) ResNet50V2 and (b) VGG-16 models without using weight fusion.

**Figure 6:** Validation accuracy of ResNet50V2 (for the last 11 epochs) using different averaging techniques for the parameter (weight) fusion.

**Figure 7:** ROC curves for multiple classes (COVID-19, normal, and other pneumonia) using various models: (a) ResNet50V2; (b) VGG-16; (c) InceptionV3.

**Figure 8:** Feature representation based on predicted labels with t-SNE plot for multilabel classification using all base CNN models: (a) ResNet50V2; (b) VGG-16; (c) InceptionV3.

**Figure 9:** Model interpretation with heatmap visualization using Grad-CAM for (a) COVID-19 patients, model: ResNet50V2; (b) COVID-19 patients, model: InceptionV3; (c) pneumonia patients, model: ResNet50V2.

**Table 1:** Training, validation, and test datasets from various CXR image categories.

Class	No. of samples			
	Training set (60%)	Validation set (20%)	Testing set (20%)	Total (100%)
Normal	368	124	124	616
Pneumonia	368	124	124	616
COVID-19	368	124	124	616

**Table 2:** Parameters and functions used for model training.

Training parameters	Values/types
Epoch count	50
Size of batch	8
Optimizer	Adam
Loss function	Categorical cross-entropy
Warmup learning rate	0.001
Rotation range	15
Shear range	10%
Zoom range	10%
Width and height shifting	10%
Horizontal flip	Yes
Fill mode	Nearest
Rescaling	1/255

**Table 3:** Classification results for ResNet50V2, VGG-16, and InceptionV3 on the holdout test dataset.

Model	Accuracy	Precision	Sensitivity	Specificity	F1-score	AUC
ResNet50V2	95.49	96.85	99.19	98.27	98.00	95.94
VGG-16	92.70	97.50	94.35	98.69	95.89	95.73
InceptionV3	92.97	97.60	98.39	98.67	97.99	94.72

**Table 4:** Performance results for each class using all evaluated models on the test dataset.

Model	Class	Accuracy	Precision	Recall	F1-score
ResNet50V2	Pneumonia	90.24	93.0	90.0	92.0
	Normal	94.30	94.0	94.0	94.0
	COVID-19	99.19	97.0	99.0	98.0

VGG-16	Pneumonia	89.43	90.0	89.0	90.0
	Normal	94.30	91.0	94.0	92.0
	COVID-19	94.35	97.0	94.0	96.0

InceptionV3	Pneumonia	86.99	91.0	87.0	89.0
	Normal	93.49	90.0	93.0	92.0
	COVID-19	98.38	98.0	98.0	98.0

**Table 5:** Confusion matrix for COVID-19 class using the test dataset.

Model	TP	FP	TN	FN
ResNet50V2	123	4	227	1
VGG-16	117	3	226	7
InceptionV3	122	3	222	2

**Table 6:** Comparison of the proposed weight fusion model with other existing deep learning-based studies from the literature.

Method	Target classes	Evaluation results				
		Acc.	Prec.	Sens.	Spec.	AUC
Proposed fusion method	3 classes: COVID-19, normal, pneumonia	0.954	0.968	0.991	0.982	0.959
COVID-Net [31]	3 classes: COVID-19, normal, non-COVID-19	0.933	0.989	0.910	—	—
CovidGAN [25]	2 classes: COVID-19, normal	0.950		0.900	0.970	—
Pretrained CNN [17]	2 classes: COVID-19, normal	0.980	1.00	0.960	1.00	—
ResNet18 [18]	5 classes: normal, bacterial, tuberculosis, viral, COVID-19	0.889	0.834	0.859	0.964	—
Triple-view CNN [15]	2 classes: normal, COVID-19	0.998	0.996	0.999	0.997	—
	3 classes: normal, COVID-19, other	0.844				
DarkNet [19]	2 classes: COVID-19, no findings	0.980	0.980	0.951	0.953	—
	3 classes: COVID-19, no findings, pneumonia	0.870	0.899	0.853	0.921	—
Deep learning-based decision tree [21]	Multiple classes: COVID-19, TB, non-COVID-19, non-TB	0.950	0.940	0.970	0.930	0.950

## Data Availability

The CXR images used in this study are collected from two open-source data repositories: 1. https://github.com/ieee8023/covid-chestxray-dataset; 2. https://www.kaggle.com/paultimothymooney/chest-xray-pneumonia.
